# Tobacco Use and Its Associated Factors among Undergraduate Public Health Students in Kathmandu Valley, Nepal

**DOI:** 10.1155/2022/1495779

**Published:** 2022-07-08

**Authors:** Birendra Chand, Sandesh Bhusal, Pranil Man Singh Pradhan, Kiran Paudel, Nisha Adhikari, Tara Ballav Adhikari, Sushan Man Shrestha

**Affiliations:** ^1^Institute of Medicine, Tribhuvan University, Kathmandu, Nepal; ^2^Nepal Health Frontiers, Tokha-5, Kathmandu, Nepal; ^3^Department of Community Medicine, Maharajgunj Medical Campus, Institute of Medicine, Tribhuvan University, Kathmandu, Nepal; ^4^Section for Global Health, Department of Public Health, Aarhus University, Aarhus, Denmark; ^5^COBIN Project, Nepal Development Society, Bharatpur 10, Chitwan, Nepal

## Abstract

**Background:**

Despite the crucial role of public health students in tobacco control, there is a paucity of information regarding tobacco use among this population in Nepal. This study aims to assess the prevalence of tobacco use among undergraduate public health students in Kathmandu valley, Nepal.

**Methods:**

A web-based survey was conducted among 386 undergraduate public health students in Kathmandu valley, Nepal, using the Global Health Professions Student Survey (GHPSS) questionnaire. Associated factors were examined using multivariate logistic regression analyses at the level of significance of 0.05.

**Results:**

A total of 16.8% of students were current cigarette smokers, 39.9% had ever smoked cigarettes, and 62.2% had smoked their first cigarettes during adolescence. Among the participants, 11.7% currently used other tobacco products. Male students (aOR: 15.4; 95% CI: 4.9–47.8), students with higher age (aOR: 2.4; 95% CI: 1.0–5.4), students belonging to non-Brahmin/Chhetri ethnic group (aOR: 2.3; 95% CI: 1.2–4.4), and those staying without family (aOR: 2.0; 95% CI: 1.1–5.0) had higher odds of being current smoker. Similarly, students with a parental history of tobacco use (aOR: 2.4; 95% CI: 1.3–5.0) and friends with smoking habits (aOR: 7.9; 95% CI: 2.3–27.0) were more likely to be a current smoker.

**Conclusion:**

There is a notable prevalence of tobacco use among public health students in Kathmandu valley, Nepal. Concerned stakeholders should work jointly to implement a cessation program to discourage tobacco use among these populations who have a potential role in educating communities about the hazards of tobacco smoking, tobacco use prevention, and control.

## 1. Introduction

The tobacco epidemic is one of the biggest public health threats the world has ever faced, killing more than 8 million people a year globally. More than 7 million of those deaths result from direct tobacco use, while around 1.2 million are the result of nonsmokers being exposed to second-hand smoke [1]. Tobacco use is the leading global cause of preventable death [2] and a major proven risk factor contributing substantially to the rising burden of noncommunicable diseases [3].

In South Asia, approximately 1.2 million people die yearly from tobacco consumption. Although Bangladesh, Nepal, and Sri Lanka have country-specific tobacco control laws and policies, tobacco consumption among the youths is common, and the magnitude of the problem is increasing [4]. The WHO STEPwise Approach to NCD Risk Factor Surveillance (WHO-STEPS survey) Nepal 2019 showed that 28.9% of adults aged 15–69 years currently used either smoked tobacco or smokeless tobacco products. Despite adopting tobacco control laws and policies, there has been no significant reduction in tobacco users between 2013 and 2019 in Nepal [5].

It has been estimated that 70% of premature deaths among adults are due to behavioral patterns that emerge in adolescence; including smoking, violence, and sexual behavior [6]. The undergraduate stage is crucial as it is the transition period from teenager to young adult, moving out of home and relying less on parents to make daily life decisions. It is usually seen that risk-taking behaviors begin to manifest during this stage [3, 6–8]. Also, college students are easy targets for the tobacco industry; young people like them are bombarded with protobacco messages and sometimes offered free tobacco products [8]. The WHO Framework Convention on Tobacco Control (FCTC) emphasizes the vital contribution of participation of health professional bodies, training, and healthcare institutions in tobacco control efforts. Health professionals who smoke also send an ambiguous message to patients they have encouraged to cease smoking [9].

Future public health professionals have a leading role in combating smoking in the community. They play a significant role in educating communities about the hazards of tobacco smoking, tobacco use prevention, control, and cessation efforts. However, studies have shown that health professionals who smoke cannot be expected to persuade patients and community people to quit smoking [10, 11]. Thus, it is essential to determine their tobacco consumption pattern before implementing any antitobacco measures.

Despite the crucial role of public health professional students in tobacco control, very few studies have collected information regarding the use of tobacco, exposure to second-hand smoke, and tobacco cessation among public health students in Nepal. Therefore, this study aimed to assess the prevalence of tobacco use and its associated factors, second-hand smoke exposure, and behavior related to tobacco cessation among public health students in Kathmandu valley.

## 2. Methods

### 2.1. Study Setting

The study was conducted in the public health colleges under Tribhuvan University, Pokhara University, and Purbanchal University, located inside the Kathmandu Valley, Nepal.

The Kathmandu valley consists of three districts: Kathmandu, Bhaktapur, and Lalitpur, and most of the public health colleges affiliated with the three universities are located inside the Kathmandu valley. A majority of undergraduate public health students have been pursuing their education on these campuses.

### 2.2. Study Population

The study population was public health students pursuing undergraduate degrees under the colleges of Tribhuvan University, Pokhara University, and Purbanchal University, located inside the Kathmandu Valley, Nepal. Undergraduate public health students from the first academic year to the fourth academic year (last), studying under three universities inside Kathmandu valley, were eligible for selection.

### 2.3. Study Design and Sample

This was a web-based descriptive cross-sectional study conducted between January and February 2021. The expected prevalence of tobacco use in the population was taken as 29% from the STEPS Survey Nepal, 2019 [5], and the sample size was calculated using the Cochran's formula; *n* = *z*^2^pq/*e*^2^, where *p*=0.29, , *q* = 0.71, *z* = 1.96 at 95% confidence interval, and *e* = 0.05.

Therefore, the calculated sample size was 316, and considering the 20% nonresponse rate, the sample size obtained was 395. The convenient sampling technique was employed to select the participants.

### 2.4. Data Collection Methods

Online questionnaires on online Google forms were administered via e-mail and social media platforms to collect data from the participants. Study participants were encouraged to complete the online survey form at their convenience. Single response from each student was ensured via Google Forms setting by choosing “Limit to 1 response.”

### 2.5. Measurements

#### 2.5.1. Smoking Status

A self-administered validated Global Health Professions Student Survey (GHPSS) questionnaire, a validated tool for screening smoking among university students [12], was used for this study, which was developed by the World Health Organization (WHO), the US Centers for Disease Control and Prevention (CDC), and the Canadian Public Health Association [13].

 
*Current smoker* is defined as one who had smoked cigarettes daily or occasionally during the past 30 days preceding the survey.
 
*Nonsmoker* is defined as one who had never smoked a cigarette in their lifetime.
 
*Ever smoker* is defined as one who had smoked even a single cigarette in their lifetime.
 
*Other tobacco products* are chewing tobacco, snuff, bidis, hookah, cigar, or pipes.

### 2.6. Explanatory Variables

Explanatory variables were age, sex, family type (nuclear, joint/extended), ethnicity (categorized as Brahmin/Chhetri, Janajati, Madhesi, Muslim, Dalit, and others according to Health management information system, Nepal government)[14], place of residence (categorized as rural and urban), current residence status (staying with/without family) [15], parental history of tobacco use (yes/no), and friends with tobacco using habit (yes/no).

### 2.7. Data Analysis

Statistical analysis was performed using IBM SPSS version 20. Descriptive analysis was done by calculating frequency and percentages for categorical variables and mean and standard deviation for continuous variables. The association between categorical independent variables and categorical dependent variables was measured by the Chi-square test followed by binary logistic regression analyses.

### 2.8. Ethical Consideration

Ethical clearance was obtained from the Institutional Review Committee (IRC) of the Institute of Medicine (IOM) (ref. no.: 215 (6–11) *E*^2^077/078). All the participants were informed about the aims and objectives of the study by including the electronic consent form in the Google form questionnaire. The participants were aware that their participation was voluntary. The confidentiality of the participants was ensured.

## 3. Results

### 3.1. Study Participant Characteristics

Table 1 illustrates the characteristics of the study participants. A total of 386 participants were eligible for analysis. The mean age (±SD) of the participants was 22 (±2.2) years. Almost similar proportions of males (49.0%) and females (51.0%) participated in the study. Brahmin/Chhetri was the predominant ethnic group (61.9%) followed by Janajati (20.5%). Higher proportions of participants were from the nuclear family (70.7%). Around 60% of the participants were currently staying with their families.

### 3.2. Prevalence of Tobacco Use

A total of 16.8% of students were current cigarette smokers. More than one-third of the total participants had smoked cigarettes ever (39.9%), and the majority of them (62.2%) had smoked their first cigarette during their adolescence life (11–19 years). A total of 11.7% of participants currently used other tobacco products like chewing tobacco, snuff, bidis, hookah, cigar, or pipes, and 28.8% had ever tried other tobacco products (Table 2).

### 3.3. Exposure to Tobacco Smoke

Among the total participants, 17.9% were exposed to second-hand smoke at home during the last week preceding the survey. The proportion was higher among males (72.5%) compared to females (27.5%). Similarly, 41.5% of the participants were exposed to second-hand smoke at public places during the past week preceding the survey (Table 3).

### 3.4. Behavior Related to Tobacco Cessation

Table 4 shows behaviors related to tobacco cessation among study participants. Among the current smokers (*n* = 65), 47.7% want to stop smoking cigarettes now, 52.3% had ever tried to stop smoking cigarettes, and 73.8% of them had ever received help or advice to stop smoking cigarettes.

### 3.5. Association of Smoking with Independent Variables

There was a significant association between the age of the participants and smoking status. Higher age groups (aOR: 2.4, 95% CI: 1.0–5.4) were more likely to be current smokers than lower age groups. Male participants were 15.4 (95% CI: 4.9–47.8) times more likely to be current smokers as compared to females. Participants belonging to the non-Brahmin/Chhetri group were almost twice more likely to be a current smoker than the Brahmin/Chhetri group (aOR: 2.3, 95% CI: 1.2–4.4). Compared to participants who stayed with their family, participants who stayed alone/with friends were two times more likely to be current smokers (aOR: 2.0, 95% CI: 1.1–5.0). Similarly, participants who reported a history of tobacco use in their family were 2.4 times more likely to be a current smoker than those with no previous history of tobacco use in their family (95% CI: 1.3–5.0). Participants who have friends with habits of tobacco use had more odds of being current smokers than those who did not have friends who used tobacco (aOR: 7.9, 95% CI: 2.3–27.0) (Table 5).

## 4. Discussion

In this study, the prevalence of current smokers was found to be 16.8% which is similar to the prevalence reported in a study conducted among Nepalese health professional students [16]. This prevalence rate is lower than the general population (33.0%) and higher than the 15–19- year-old adolescents (15.8%) at the national level [17]. The prevalence of ever smokers was 39.9% which is lower than a similar study conducted among medical students in Kathmandu, Nepal. However, this rate is higher than the study conducted among health professional students in Chitwan, Nepal [16].

The prevalence of current other tobacco products such as chewing tobacco, sniffs, bidis, hookah, cigars, and pipes is 11.7% which is higher than the prevalence reported in several studies conducted across Nepal and India among health professional students [12, 16, 18].

Most students initiated smoking during their adolescent stage (11–19 years). Studies conducted in Nepal [3, 16, 19] and India [20] have shown a similar smoking initiation pattern. Early- and middle-adolescents are more vulnerable to initiation of risk-taking behavior like tobacco use and smoking. Factors such as curiosity, relieving tension, and pressure from friends might be the reasons for initiating smoking at earlier/younger age [3].

Higher odds of being a current smoker were found in the students with a higher age group (>21 years). This is in contrast to the study conducted among university health science students in Lao People's Democratic Republic (Lao PDR) [9] where no significant difference in the smoking pattern was observed between age groups. Students of higher age might be living independently far from their families and might have received higher pocket money. These factors could have made tobacco products more accessible to them.

There was a striking difference in smoking between males (15.3%) and females (1.5%) in our study. Males were more likely to be a current smoker as compared to females. Studies conducted among health professional students in Nepal [12], China [21], and Lao PDR [9] have reported similar findings. Smoking can be considered as part of a constellation of risk-taking behaviors that are more prevalent among men. In the context of Nepal, smoking is viewed as acceptable behavior for boys but not for girls, especially among the unmarried [3]. Non-Brahmin/Chhetri ethnic groups have higher odds of being current smokers as compared to Brahmin/Chhetri in our study. The attitude towards smoking is more permissive among the people belonging to the non-Brahmin/Chhetri ethnic group [3]. This might be a possible explanation for the higher odds of smoking seen among the non-Brahmin/Chhetri.

Studies from India and Nepal have mentioned the influence of family type on tobacco use [3, 6]. However, in our study, smoking status was not associated with family type. This difference might be due to the difference in sampling size of the studies. Compared to students staying with their family, participants staying alone/with friends were more likely to be current smokers. This contrasts with the findings from a study conducted among junior collegiate in western Nepal [22], where no association was observed between smoking status and current residential status. Close contact among parents and children might have played a protective role against taking up risky behavior like smoking among students who were staying with their families.

Our study revealed that current smoking was significantly associated with parental history of tobacco use which is consistent with a study conducted among Chinese students [23]. A study conducted in western Nepal also showed that, as the number of family members using tobacco increased by a unit, the risk of tobacco use increased by 1.5 times [22].

In our study, students who have friends with tobacco using habits were almost eight times more likely to be current smokers. Several studies have mentioned peer pressure and friends' influence on smoking behavior [24–26]. Smoking behavior is related to the behaviors of their friends and parents. There are several ways in which friends can influence cigarette use, such as through the modeling of risky behaviors and normative peer pressures [27]. A review conducted by Hoffman et al. has mentioned that the number of friends who smoke is the most common risk factor linked to cigarette use and a stronger predictor than other peer influence measures [28].

### 4.1. Study Limitations

The present study had a few limitations. All the measurements in this study were based on self-reports, which may have been prone to response and information bias. There might have been the introduction of selection bias as those students without reliable Internet access might not have participated in the study. The cross-sectional study design could not establish the temporal association between the independent variables and tobacco use.

To the best of our knowledge, this is the first study exploring tobacco consumption and smoking patterns among Nepalese public health students. Despite limitations, this study provided information regarding tobacco use and smoking among the less explored population in Nepal. The findings of this study added evidence to the limited literature on tobacco consumption among health professional students in Nepal.

## 5. Conclusion

This study reported a notable prevalence of smoking and use of other tobacco products among public health students in Kathmandu valley, Nepal. The cigarette is the most commonly used tobacco product than any other form of tobacco. We urge concerned stakeholders to take measures to discourage tobacco use among health profession undergraduate students who are considered to play a significant role in educating communities about the hazards of tobacco smoking, tobacco use prevention, control, and cessation efforts. Legislations on the use of tobacco products need to be enforced to decrease the availability, accessibility, and affordability of tobacco products.

## Figures and Tables

**Table 1:** Study Participants characteristics.

Characteristics	Number (%)
Age group (years)	
≤21 years	152 (39.4)
>21 years	234 (60.6)

Sex	
Male	189 (49)
Female	197 (51)

Religion	
Hinduism	367 (95.1)
Buddhism	8 (2.1)
Christianity	9 (2.3)
Islam	2 (0.5)

Ethnicity	
Brahmin/chhetri	239 (61.9)
Janajati	79 (20.5)
Madhesi	41 (10.6)
Dalit	11 (2.8)
Others	16 (4.1)

Family type	
Nuclear	273 (70.7)
Joint/extended	113 (29.3)

Permanent residence	
Urban	194 (50.3)
Rural	192 (49.7)

Current residence	
Staying alone	77 (19.9)
Staying with friends	77 (19.9)
Staying with family	232 (60.1)

Parental history of tobacco use	
Yes	150 (38.9)
No	236 (61.1)

Friends with tobacco using habit	
Yes	233 (60.4)
No	153 (39.6)

University	
Tribhuvan	142 (36.8)
Pokhara	113 (29.3)
Purbanchal	131 (33.9)

Academic year	
First	79 (20.5)
Second	89 (23.1)
Third	109 (28.2)
Fourth	109 (28.2)
Total	**386 (100)**

**Table 2:** Prevalence of tobacco use (*n* = 386).

Characteristics	Male (%)	Female (%)	Total (%)
Ever tried/experimented with cigarette smoking			
Ever tried	116 (75.3)	38 (24.7)	154 (39.9)
Never tried	75 (31.9)	158 (68.1)	232 (60.1)

Respondent's age when initiated smoking			
≤10 years	15 (54.6)	7 (45.4)	22 (8.4)
11–19 years	80 (77.9)	25 (22.1)	105 (62.2)
≥20 years	32 (63.7)	16 (36.3)	48 (25.4)

Current smoking status			
Current smoker	61 (93.8)	4 (6.2)	65 (16.8)
Current nonsmoker	128 (39)	193 (60.1)	321 (83.2)

Ever tried other tobacco products			
Ever tried	74 (66.7)	37 (33.3)	111 (28.8)
Never tried	115 (41.8)	160 (58.2)	275 (71.2%)

Currently using other tobacco products			
Current user	33 (73.3)	12 (26.7)	45 (11.7)
Current nonuser	156 (45.7)	185 (54.3)	341 (88.3)
Total	**189 (100)**	**197 (100)**	**386 (100)**

**Table 3:** Exposure to tobacco smoke.

Characteristics	Male (%)	Female (%)	Total (%)
Exposure to tobacco smoke at home during the past week			
Exposed	50 (72.5)	19 (27.5)	69 (17.9)
Nonexposed	139 (43.8)	178 (56.2)	317 (82.1)

Exposure to tobacco smoke at public places during the past week			
Exposed	99 (61.9)	61 (38.1)	160 (41.5)
Nonexposed	90 (39.8)	136 (60.2)	226 (58.5)
Total	**189 (100)**	**197 (100)**	**386 (100)**

**Table 4:** Behavior related to tobacco cessation.

Behaviors	Number (%)
Wanting to stop smoking cigarettes now	31 (47.7)
Ever tried to stop smoking cigarettes	34 (52.3)
Ever received help or advice to stop smoking cigarettes	48 (73.8)

**Table 5:** Association of smoking with independent variables.

Variables	Smoking status		Unadjusted odds ratio (95% CI)	Adjusted odds ratio (95% CI)
	Current smoker (%)	Not current smoker (%)		
Age				
>21 years	48 (20.5)	186 (79.5)	2.1 (1.1–3.7)^*∗*^	2.4 (1.0–5.4)^*∗*^
≤21 years (ref)	17 (11.2)	135 (88.8)	1	1

Sex				
Male	61(32.3)	128 (67.7)	22.9 (8.2–64.8)^*∗∗*^	15.4 (4.9–47.8)^*∗∗*^
Female (ref)	4 (2.0)	193 (98.0)	1	1

Ethnicity				
Non-Brahmin/Chhetri	34 (23.1)	113 (76.9)	2.0 (1.2–3.5)^*∗*^	2.3 (1.2–4.4)^*∗*^
Brahmin/Chhetri (ref)	31 (13.0)	208 (87.0)	1	1

Family type				
Nuclear	41 (15.0)	232 (85.0)	0.6 (0.4–1.1)	0.7 (0.4–1.5)
Joint/extended (ref)	24 (21.2)	89 (78.8)	1	1

Permanent residence				
Rural	41 (21.4)	151 (78.6)	1.9 (1.1–3.3)^*∗*^	0.9 (0.4–1.8)
Urban (ref)	24 (12.4)	170 (87.6)		

Current residence				
Staying without family	27 (17.5)	127 (82.5)	1.1 (0.6–1.9)	2.0 (1.1–5.0)^*∗*^
Staying with family (ref)	38 (16.4)	194 (83.6)	1	1

Academic year				
Higher year	33 (15.1)	185 (84.9)	1.4 (0.76–2.5)	0.8 (0.4–1.7)
Lower year (ref)	32 (19.0)	136 (81.0)	1	1

Parental history of tobacco use				
Yes	38 (25.3)	112 (74.7)	2.6 (1.5–4.5)^*∗∗*^	2.4 (1.3–5.0)^*∗*^
No (ref)	27 (11.4)	209 (88.6)	1	1

Friends with tobacco using habit				
Yes	62 (26.6)	171 (73.4)	18.1 (5.6–58.9)^*∗∗*^	7.9 (2.3–27.0)^*∗∗*^
No (ref)	3 (2.0)	150 (98.0)	1	1

Note: ^*∗*^ = *p* value less than 0.05. ^*∗∗*^ = *p* value less than 0.001.

## Data Availability

Data are available on reasonable request to the corresponding author.

## Abbreviations

AOR: Adjusted odds ratio
CDC: Centers for Disease Control and Prevention
CI: Confidence interval
GHPSS: Global Health Professions Student Survey
Lao PDR: Lao People's Democratic Republic
SD: Standard deviation
WHO: World Health Organization.
